# Micro Learning Support Vector Machine for Pattern Classification: A High-Speed Algorithm

**DOI:** 10.1155/2022/4707637

**Published:** 2022-08-03

**Authors:** Yu Yan, Yiming Wang, Yiming Lei

**Affiliations:** ^1^School of Economics, Peking University, Haidian District, Beijing 100871, China; ^2^Key Laboratory of Mathematical Economics and Quantitative Finance, Peking University, Haidian District, Beijing 100871, China

## Abstract

The support vector machine theory has been developed into a very mature system at present. The original support vector machine to solve the optimization problem is transformed into a direct calculation formula of line in this paper and the model is *o*(*n*^2^) time complexity. In the model of this article, weited theory, multiclassification problem and online learning have all become the direct inference, and we have applied the new model to the UCI data set. We hope that in the future, this model will be useful in real-world problems such as stock forecasting, which require nonlinear hi-speed algorithms.

## 1. Introduction

Since the establishment of the support vector machine ([1–3]) in 1995, Vapnik et al., the support vector machine(SVM) has been the focus of researchers in data mining. The classical SVM processing is a classic binary classification problem, where SVM labels unlabeled points by solving an optimal line. One of the basic principles of SVM is to use kernel technology so that the specific mapping method cannot be known. Throu the simple inner product of the nonlinear problem in the original space, we can solve this problem with a linear problem in another space that is mapped to. Moreover, the model can significantly improve the time complexity of the small sample problems throu dual theory, and one of the classic model thinking: the maximum interval is also widely used in various models^1^.

In 2007, Jayadeva et al. ([4–7]) established the model as the twin support vector machine (TWSVM), which solves the classic two classification problem. Unlike SVM, TWSVM is mainly used to solve nonparallel problems. The support surface of the SVM is two parallel hyperplanes, and TWSVM is the solution to the two nonparallel hyperplanes. This model no longer uses the maximum interval principle in SVM. TWSVM solves for two straight lines that are as close as possible to the two classes of points. Classification is performed by determining which line a new point is close to.

SVM has a time complexity of *o*(*n*^3^+*d*) when the number of samples is *n* and the number of characteristics is *d*, making SVM very suitable for solving hi-dimensional small sample problems. Some other algorithms are also suitable for small samples, but they have mutual advantages and disadvantages with SVM^2^. The kernel technique also makes SVM very suitable for solving nonlinear problems and hi-dimensional problems. There are also some algorithms that are suitable for hi-dimensional problem, but they have mutual advantages and disadvantages with SVM^3^. However, a common problem with a range of algorithms based on SVM is the inability to solve large-sample problems due to the limitations of the optimization algorithm. Therefore, we want to provide algorithm that maintains the good properties of SVM while reducing the time required to solve large sample sizes. We give a nonoptimal SVM model with a time complexity of *o*(*n*^2^+*d*). This improvement will go some way towards circumventing the problem that SVM cannot be applied to large-scale data. Our model can be applied to many hi-dimensional or large sample problems^4^ and has substantial implications for solving real-world problems with hi-dimensional, large samples, and hi-time demands.

In this paper, we consider a kind of nonoptimal machine learning model from the point of view that there is only one positive and one negative. The model takes a point from the positive and negative points to train a model, and then uses all the combinations of positive and negative points. Finally, the model is considered by using multiple models.

The basic logic of the model is that it can be used to train several classification models. In this case, we construct a classification model which can be used in kernel technology. It is interesting to note that in this model, the problems of machine learning, such as the classification problem, the weited problem, and the fitting problem, will be straitforward to operate.

The details of our research are shown in Figure 1.

## 2. Classical Model

Consider the classic two classification problem: given training set (*x*_*i*_, *y*_*i*_) ∈ ℝ^*d*^ × {−1,1}, *i* = 1,2,3,…, *n* where *y*_*i*_ is the label, and we have to look for the decision function *f*(*x*) to infer any new input *x* corresponding output *y*. In order to facilitate the representation, we use the following notation: *A* represents a data set of positive class points, and *B* represents the data set of negative class points.

First, we review the classical linear SVM model. The model aims to establish a strait line between positive and negative, two types of samples. One of the principles of SVM is the principle of maximum distance, that is, to maximize the distance between two support planes. We assume that the dividing surface is *wx*+*b*=0, and the two support surface is *wx*+*b*=1 and *wx*+*b*=−1. The problem of solving the problem of SVM is changed into the following optimization problem:

(1) $$\begin{array}{c} \text{min}\frac{1}{2}{\left\|w\right\|}^{2},\\ s.t.y_{i}\left(wx_{i}+b\right)\geq 1. \end{array}$$

On the other hand, the linear optimization problem is as follows:

(2) $$\begin{array}{c} \min\frac{1}{2}{\left\|w\right\|}^{2},\\ s.t.y_{i}\left(wx_{i}+b\right)\geq 1,\\ q_{i}\geq 0. \end{array}$$

Then, we consider the kernel technology in the dual problem and transform *x*_*i*_*x*_*j*_ into *K*(*x*_*i*_, *x*_*j*_). The Euclidean space is mapped into another space, and the nonlinear problem is transformed into a linearly separable problem in a hi-dimensional space.

We look back on another machine learning algorithm: the TWSVM. The TWSVM focuses on solving the nonparallel problem. Two types of sample points are enriched near the two parallel lines. The model aims to find two nonparallel strait lines, which can be used to determine the type of line in the classification. The optimization problem of the model is as follows:

(3) $$\begin{array}{c} \left(\text{TWSVM}1\right)\text{Min}\frac{1}{2}{\left(Aw_{1}+b_{1}\right)}^{T}\left(Aw_{1}+b_{1}\right)+c_{1}e_{2}^{T}bq_{1}\\ s.t.-{\left(Bw_{1}+b_{1}\right)}^{T}+q\geq e_{2},q\geq 0,\\ \left(\text{TWSVM}2\right)\text{Min}\frac{1}{2}{\left(Bw_{2}+b_{2}\right)}^{T}\left(Bw_{2}+b_{2}\right)+c_{2}e_{1}^{T}bq_{2}\\ s.t.{\left(Aw_{2}+b_{2}\right)}^{T}+q\geq e_{1},q\geq 0. \end{array}$$

The dual problem of the model is as follows:

(4) $$\begin{array}{c} \left(\text{DTWSVM}1\right){\text{Maxe}}_{2}^{T}\alpha -\frac{1}{2\alpha^{T}}G\left(H^{T}H\right)G^{T}\alpha \\ s.t.0\leq \alpha \leq c_{1},\\ \left(\text{DTWSVM}2\right){\text{Maxe}}_{1}^{T}\gamma -\frac{1}{2\gamma^{T}}H\left(G^{T}G\right)H^{T}\gamma \\ s.t.0\leq \gamma \leq c_{2}, \end{array}$$

where *H*=[*A*, *e*1] and *G*=[*B*, *e*2].

In order to introduce kernel technology, we consider replacing the two strait lines *xw*^1^+*b*^1^=0 and *xw*^2^+*b*^2^=0 (*X* is the sum of *A* and *B*).

(5) $$\begin{array}{c} k\left(x,X\right)w_{1}+b_{1}=0,\\ k\left(x,X\right)w_{2}+b_{2}=0. \end{array}$$

The dual problem is as follows:

(6) $$\begin{array}{c} \left(\text{KDTWSVM}1\right){\text{Maxe}}_{2}^{T}\alpha -\frac{1}{2\alpha^{T}}R\left(S^{T}S\right)R^{T}\alpha \\ s.t. 0\leq \alpha \leq c_{1},\\ \left(\text{KDTWSVM}2\right){\text{Maxe}}_{1}^{T}\gamma -\frac{1}{2\gamma^{T}}S\left(R^{T}R\right)S^{T}\gamma \\ s.t. 0\leq \gamma \leq c_{2}, \end{array}$$

where *S*=[*k*(*A*, *X*^*T*^), *e*1] and *R*=[*k*(*B*, *X*^*T*^), *e*2];

## 3. New Model

Firstly, we consider the process of learning. If we only have a sample point, for example, if our problem is how to determine whether a person is male or female and the training set is just a lady in the picture. Then, we cannot judge another picture of the characters in the male and female. It is difficult to classification when we have only one class of points. By the same token, even thou our training focuses on ten thousand women's photographs, without a single photo of men, it is still unable to train a model that can distinguish between men and women. It is difficult for us to compare the difference between a man and ten thousand women in our normal human thinking, and we can only compare the difference between a male and a female.

Therefore, we consider a positive point and a negative point. The training set has only one positive and one negative point. Using the idea of the maximum interval of SVM, we can obtain that the optimal line is the two points of the vertical bisector of the line, and the functional distance between the two points and a strait line is 1 in Figure 2.

Obviously, we can get the dividing line as follows:

(7) $$\begin{array}{c} \frac{2\left(x^{+}-x^{-}\right)x}{{\left(x^{+}-x^{-}\right)}^{2}}-\frac{{\left(x^{+}\right)}^{2}-{\left(x^{-}\right)}^{2}}{{\left(x^{+}-x^{-}\right)}^{2}}=0. \end{array}$$

Then, we consider a very interesting classification problem, as shown in figure two in Figure 3.

From Figure 3, we can see that each point in the positive point and negative point in the class make the points of the line, and finally, the combination of points is a reasonable way. So we consider the following algorithm.

Then, we consider the general situation, that is, the number of positive and negative points (in order to facilitate the consideration, we assume that there are *M* positive points and *N* negative points). Take a positive point and a negative class point, and we can get its vertical bisector.

(8) $$\begin{array}{c} \frac{2\left(x^{+}-x^{-}\right)x}{{\left(x^{+}-x^{-}\right)}^{2}}-\frac{{\left(x^{+}\right)}^{2}-{\left(x^{-}\right)}^{2}}{{\left(x^{+}-x^{-}\right)}^{2}}=0. \end{array}$$

We consider the calculation of all the points, and then use each of the subline to consider the classification problem.

The core idea of this algorithm is to take each positive point and each negative class point out to build a subline, and then all the points out of an average. Take the positive and negative values as the classification results and we consider the classification results are as follows:

(9) $$\begin{array}{c} \text{sign}\left(\sum_{i=1}^{m}\sum_{j=1}^{n}\frac{2\left(x^{i}-x^{j}\right)x}{{\left(x^{i}-x^{j}\right)}^{2}}-\frac{{\left(x^{i}\right)}^{2}-{\left(x^{j}\right)}^{2}}{{\left(x^{i}-x^{j}\right)}^{2}}\right). \end{array}$$

After we discuss an improvement of the model, we consider the following sample points in Figure 4.

In the training of the sample points, if we consider the model we calculate, it will lead to the left side of the figure, resulting in the training model is not reasonable. The foundation of our model is the two point training division. We consider the linear translation, namely, the introduction of a parameter *C* in(−1,1) two, making the line training as follows:

(10) $$\begin{array}{c} \text{sign}\left(\sum_{i=1}^{m}\sum_{j=1}^{n}\frac{2\left(x^{i}-x^{j}\right)x}{{\left(x^{i}-x^{j}\right)}^{2}}-\frac{{\left(x^{i}\right)}^{2}-{\left(x^{j}\right)}^{2}}{{\left(x^{i}-x^{j}\right)}^{2}}+\text{Cmn}\right). \end{array}$$

Then, we introduce the nucleus to each line. Since our model is only composed of the inner product of two vectors, we can use *K*(*x*, *y*) to replace the *xy*, which can be obtained as follows:

(11) $$\begin{array}{c} \text{sign}\left(\sum_{i=1}^{m}\sum_{j=1}^{n}\frac{2\left(K\left(x^{i},x\right)-K\left(x^{j},x\right)\right)}{K\left(\left(x^{i}-x^{j}\right),\left(x^{i}-x^{j}\right)\right)}-\frac{K\left(x^{i},x^{i}\right)-K\left(x^{j},x^{j}\right)}{K\left(x^{i}-x^{j},x^{i}-x^{j}\right)}+\text{Cmn}\right). \end{array}$$

It is evident that the time complexity of the model is *O*(*n*^2^). Because we have a large number of points to get the average score, the weited sum of the sample points is the direct inference of the model. Similarly, if we want to get an online learning model or give up some of the sample points, the time complexity will be very low. Under this premise, the training complexity of the multiclassification problem is also very low.

## 4. Data Testing

First, we compute the linear kernel on the UCI dataset, and the accuracy and variance contrast is shown in Table 1.

We can see that the new model has a good advantage, and then we consider the computation of the nonlinear RBF kernel on the UCI data set in Table 2.

In the theory, we show that the new algorithm has strong superiority in time complexity. Here, we do some experiments to count. It can be seen that there are great advantages of some data sets. Then, we calculate the computation time of the linear kernel and the nonlinear kernel on the different number of data sets in Table 3.

In addition to the analysis of the time complexity of the linear problem, we then count the time of the nonlinear case. Then, we apply the nonlinear kernel in Table 4.

The time complexity of our model is *o*(*n*^2^+*d*). The time complexity of the SVM and the TWSVM is *o*(*n*^3^+*d*). Based on Tables 3 and 4, our model is still faster than the SVM and the TWSVM, even in small sample problems with less than 1000 samples. Also, since our algorithm does not need to solve the optimization problem, the time of our algorithm is stable with respect to the growth of the number of samples. It can be expected that in large-scale samples, our algorithm will be much faster than SVM and TWSVM in computation.

## 5. Conclusion

Based on the point-to-point model, this paper establishes a micro learning support vector machine. The model is different from the traditional SVM in the way of solving it, and it is not necessary to solve the optimization problem. This makes the model have some difference with the traditional machine learning algorithm. Both neural networks and SVM are unknown time to calculate. The microlearning support vector machine is in a fixed time when the length of the orientation and the number of sample points are fixed. This is of great benefit to the stability of our design and practical applications. From the view of time complexity, the algorithm is better than SVM. Extending the micro learning support vector machine to weighted problems, multiclassification problems, and fitting problems is very simple and straightforward.

Our algorithm outperforms both SVM and TSVM in terms of model accuracy and computation time, and it also has good nonlinear generalisation due to the fact that we also use the kernel function. The computation time of this algorithm is explicit because it does not require solving an optimization problem. Overall, this algorithm is well suited to problems such as stock prediction and face recognition, which require nonlinear, hi-dimensional data, and hi computational speed.

Based on [8, 9], we can extend the model to a semisupervised problem in the future. We just have not come up with a suitable modelling idea yet. We believe that the ideas used to build our model can also be extended to the field of feature extraction in the future. And it can be applied to many related problems (e. g. [10, 11]).

We likewise believe that our model can be used to solve problems related to regression after a SVM-to-SVR-like transformation (e. g. [12–17]). Of particular interest is the fact that our algorithms are well suited for applications in the field of financial forecasting(e. g. [18–20].). The field of financial forecasting requires algorithms with controllable computation times and good performance for nonlinear problems.

In the same way as SVM, our algorithm can be used to solve multiclassification problems. We hope that other researchers will apply our algorithm to multiclassification-related problems in the future(e. g. [21–24]). It is worth noting that this algorithm can be used for face recognition(e. g. [25, 26]). Similarly, our model can be used to solve the multilabel problem(e. g. [27, 28]).

## Figures and Tables

**Figure 1:** Details of this paper.

**Figure 2:** Two-point classification.

**Figure 3:** Some-point classification.

**Figure 4:** Change of Cmn.

**Table 1:** Linear.

	NEW		SVM		TWSVM	
Australian	**0.816901**	0.083721	0.517857	0.011664	0.624101	0.129945
BUPA	0.571429	0.156057	**0.65942**	0.082409	0.082143	0.102602
Diabetes	0.508	0.470447	0.510552	0.093228	**0.67013**	0.136054
Heart disease	0.362712	0.501019	**0.762712**	0.077671	0.450847	0.481994
Heartstatlog	0.486364	0.08046	**0.771605**	0.07011	0.75	0.067215
Herman	0.73871	0.082558	**0.802419**	0.046327	0.73871	0.082558
Sonar	**0.661905**	0.221057	0.492063	0.190972	0.528571	0.227502
Teaching	0.683871	0.097844	0.741935	0	**0.825806**	0.131825
Balance	**0.889655**	0.119824	0.479885	0.099444	0.463793	0.15534
Breast	0.345985	0.113855	**0.466111**	0.054133	0	0

Bold indicates best.

**Table 2:** RBF.

	NEW		SVM		TWSVM	
Australian	0.852113	0.062461	**0.864286**	0.018443	0.848921	0.044736
BUPA	**0.642857**	0.08165	0.572464	0.062616	0.610714	0.055174
Diabetes	**0.748**	0.230911	0.698052	0.070361	0.67013	0.070895
Heart disease	**0.816949**	0.067158	0.762712	0.070565	0.674576	0.437833
Heartstatlog	**0.836364**	0.039277	0.771605	0.032075	0.759091	0.044536
Herman	0.422581	0.218011	**0.802419**	0.046327	0.680645	0.082558
Sonar	**0.590476**	0.234134	0.555556	0.062994	0.528571	0.493265
Teaching	0.729032	0.11081	0.790323	0.06843	**0.825806**	0.195687
Balance	**0.967241**	0.030111	0.817529	0.022314	0.815517	0.087618
Breast	**0.963504**	0.031817	0.959333	0.032331	0.416058	0.183863

Bold indicates best.

**Table 3:** Time of linear.

Number	New	SVM	TWSVM
100	0.031	0.109	0.312
200	0.035	1.257	0.381
300	0.052	2.606	0.518
400	0.055	4.25	0.801
500	0.293	8.371	0.864
600	0.73	12.32	1.076
700	1.169	15.672	1.745
800	1.465	24.623	2.599
900	1.871	26.34	3.695
1000	2.274	33.828	4.225

**Table 4:** Time of RBF.

Number	New	SVM	TWSVM
100	0.099	0.473	0.501
200	0.352	1.511	0.973
300	0.743	3.114	1.927
400	1.2	5.611	2.943
500	1.996	9.308	4.484
600	2.968	13.462	6.642
700	4.224	27.574	8.26
800	8.507	32.041	11.58
900	20.755	38.874	24.928
1000	23.47	47.883	28.152

## Data Availability

Data are from the UCI dataset.
